# Factors Associated with Poor Treatment Outcome among Hospitalized COVID-19 Patients in South Central, Ethiopia

**DOI:** 10.1155/2022/4551132

**Published:** 2022-02-23

**Authors:** Abdene Weya Kaso, Habtamu Endashaw Hareru, Taha Kaso, Gebi Agero

**Affiliations:** ^1^School of Public Health, Dilla University, Ethiopia; ^2^Department of Surgery, College of Health Science, Arsi University, Ethiopia; ^3^Department of Public Health, College of Health Science, Arsi University, Ethiopia

## Abstract

**Background:**

Deaths due to COVID-19 are common among the elderly, especially among individuals with underlying illnesses. The pandemic of the COVID-19 impaired the mental, psychological, and physical well-being of people admitted to hospitals. Furthermore, in underdeveloped countries, scarcity of medical equipment was a challenge to manage cases in public health facilities. Thus, understanding the epidemiology and clinical outcomes of COVID-19 patients who are receiving treatment is critical for developing effective treatments and assessing service quality. Therefore, this study is aimed at assessing the treatment outcomes and associated factors among patients affected by the COVID-19 virus.

**Method:**

We used an institutional-based retrospective cross-sectional analysis of 398 patients discharged in South Central, Ethiopia, between June 1, 2020, and July 5, 2021. Data were extracted using the data abstraction format. Data were entered, coded, and analyzed using the STATA 16 software. Bivariate and multivariate logistic regression analysis was used to assess the factors associated with poor treatment outcomes. A 95% confidence interval with adjusted odds ratio (AOR) and *p* value less than 0.05 were considered statistically significant.

**Result:**

In our study, the proportion of poor treatment outcomes was 61 (15.3%). Chronic pulmonary disease (AOR = 5.62; 95% CI: 2.49–12.70), asthma (AOR = 2.8; 95% CI: 1.17–6.67), chronic kidney disease (AOR = 4.81; 95% CI: 1.27–18.22),diabetic mellitus (AOR = 2.27; 95% CI: 1.02–5.09), HIV positive (AOR = 10.44; 95% CI: 3.0–36.35), worsening conditions (AOR = 3.73, 95% CI: 1.17–11.95), and age 55 and above years (AOR = 4.35, 95% CI: 1.30–14.60) were statistically associated with poor treatment outcomes.

**Conclusion:**

We found a significant number of patients had favourable treatment. Moreover, aging, having complicated situations at admission, and chronic illnesses such as COPD, CKD, asthma, diabetic mellitus, and HIV/AIDS participants were significantly associated with poor treatment outcomes. Therefore, critical follow–up and management of patients with underlying diseases and worsening health conditions during admission is required.

## 1. Background

Coronaviruses (CoVs) are RNA viruses that are single-stranded, encapsulated, and belong to the *Coronaviridae* family [1, 2]. They are classified as beta coronaviruses, gamma coronaviruses, and delta coronaviruses based on differences in protein sequences. The human coronaviruses (HCoV) HCoV-OC43, HCoV-229E, HCoV-NL63, and HCoVHKU1 are among the less pathogenic HCoV that cause a mild common cold or diarrhea [3]. Currently, three coronavirus infections have been identified, all of which are highly pathogenic and cause mild to severe respiratory tract disorders [4]. Among these, the recently discovered severe acute respiratory syndrome coronavirus (SARS-CoV), which was connected to a pneumonia outbreak in 2003 and had an 11 percent fatality rate, was linked to a pneumonia outbreak. The most prevalent clinical signs and symptoms of SARS-CoV were viral pneumonia, fever, chills, myalgia, and a nonproductive cough, with sore throats being less common. The virus has a two-to-seven-day incubation period [5]. The Middle East respiratory syndrome coronavirus (MERS-CoV) was first found in Saudi Arabia in 2012 and has a fatality rate of 35%. The virus has a two to fourteen-day incubation period, and symptoms include fever, shortness of breath, diarrhea, vomiting, cough, sore throat, and stomach discomfort, with a substantial number of critically ill patients requiring ICU treatment [3, 5].

The novel coronavirus (SARS-CoV-2) is a highly transmissible and dangerous virus that first appeared in Wuhan, China, in December [4, 6]. The virus is a beta coronavirus that causes human sickness and is transmitted through coughing and sneezing droplets. At room temperature, it can survive for up to six days on contaminated surfaces and objects. Infected patients experienced fever, dry cough, and shortness of breath as a result of the infection [7, 8]. The World Health Organization (WHO) declared the epidemic a global pandemic after it spread to other countries [9]. As of July 5, 2021, there had been 183,198,019 confirmed cases and 3,971,687 deaths worldwide [10]. On March 13, 2020, Ethiopia reported the first confirmed case of COVID-19. Until July 5, 2021, Ethiopia reported 276,323 confirmed cases and 4,327 deaths due to the COVID-19 outbreak [11, 12]. In hospitalized patients, the case fatality rate (CFR) was estimated to be roughly 5%, with an overall mortality rate of 0.25 percent among confirmed cases. COVID-19 infection fatality rates increased with age, and patients with underlying diseases had a higher death rate [13]. Approximately, 20% of patients admitted to the hospital had severe symptoms and were admitted to the ICU [4, 14]. The COVID-19 pandemic impaired people's emotional, psychological, and physical wellbeing while they were in hospitals [15–19]. The recent finding revealed that individual perceptions regarding a virus had a significant impact on the outcome of treatment. Moreover, medical and supportive care equipment shortages in low and middle-income countries (LMIC) hampered the treatment of illnesses in public health facilities [14]. Understanding the epidemiological and clinical results of COVID-19 patients undergoing therapy, in contrast, is critical for determining the efficacy of therapies and assessing service quality [20]. COVID-19 research has primarily concentrated on prevention measures, epidemiological inquiry, diagnosis, and therapy to date. To our knowledge, no studies have assessed the clinical outcomes and risk factors of COVID-19 patients admitted to hospitals in low-income countries, particularly Ethiopia. As a result, the goal of this study was to determine the treatment outcomes and associated characteristics among COVID-19 patients in Ethiopia's South Central region.

## 2. Method and Materials

### 2.1. Study Design, Population, and Setting

From September 1 to 15, 2021, we conducted an institutional-based retrospective cross-sectional study among hospitalized COVID-19 patients in the Arsi Zone of Ethiopia. There are 28 woredas and two town administrations in the Arsi zone. COVID-19 patients were treated in this zone at the Bokoji hospital treatment center, which is 56 kilometres from the zonal town of Assela. The study covered all COVID-19 patients who were treated between June 1, 2020, and July 5, 2021. Patients with incomplete medical records were excluded from the COVID-19.

### 2.2. Sample Size and Sampling Technique

We employed a single population proportion with a 95% confidence level, *Z*/2 = 1.96, 5% margin of error, design effect = 1.5, and the proportion of patients who had poor treatment outcomes (41%) [21]. We employed a correction formula because the number of patients discharged was fewer than 10,000, and the final sample for this study was 398 COVID-19 patient records. The treatment center was chosen using a multistage sampling technique, and the medical records of COVID-19 patients were assessed using a systematic random sample technique.

### 2.3. Study Variables and Operational Definition

In accordance with WHO and Ethiopian COVID-19 treatment and discharge protocol, we defined the final treatment outcome of patients under treatment as cured, transfer out, discharged with consent, or death [22, 23]. When patients were cured or discharged with a physician order for home-based treatment, the treatment outcome of the COVID-19 patient was considered favourable. Furthermore, if the COVID-19 patients died in the treatment center or were transferred out for further medical treatment to nearby treatment centers, the treatment outcome was rated poor. In this study, cured patients were defined as COVID-19 patients who had two consecutive negative polymerase chain reaction (PCR) results after 14 days. Moreover, patients who had positive PCR findings after 14 days in the hospital and were discharged for home-based treatment after clinical improvement were considered discharged with consent. Patients who died from any cause in the treatment facility after being hospitalized with COVID-19 were defined as death, whereas patients who were transferred out were defined as patients who were referred to nearby treatment facilities for an additional investigation related to any cause or COVID-19. The sociodemographic factors, comorbidity conditions, clinical characteristics, and status at admission were independent variables.

### 2.4. Data Collection Procedure and Quality Management

We retrieved data from patients' medical records using an abstraction format prepared for the study. Thus, data on patients' sociodemographic, admission status, intranasal oxygen use, place of care, length of stay, comorbidity status, and outcome were collected from COVID-19 medical records. After one day of training, two nurses extracted data, and the collected data were reviewed for consistency and completeness daily. The overall activities of data extraction were supervised by the principal investigator.

### 2.5. Data Analysis

The extracted data were entered, coded, cleaned, and analyzed using STATA version 16. We calculated the mean and standard deviations (SD) for continuous data and used frequency and percentage to describe categorical variables. Furthermore, to determine the factors associated with the outcome variable, bivariate logistic regression analyses with a 95 percent confidence level and crude odds ratio (COR) were performed, and variables with a *p* value less than 0.25 in the bivariate analysis were considered for multivariate logistic regression analysis. Finally, 95 percent confidence intervals with adjusted odds ratios of less than 0.05 were declared to have a significant association with the outcome variable.

### 2.6. Ethics Approval and Consent to Participate

We obtained ethical approval for this study from Arsi University. Consent to participate was waived since the study was conducted through a review of medical records. Individual patients were not subject to any hurt, and the data was not used for other purposes.

## 3. Result

### 3.1. Patient's Sociodemographic Characteristics

One hundred fifty-one (37.9%) patients were from urban areas, and 237 (59.5%) of participants were males. The majority (25.4%) of patients were above 54 years old, with a mean age of patients 39 (SD: 19.4 years) (Table 1).

### 3.2. Patients' Clinical Characteristics

Among 374 patients with clinical signs and symptoms, 82 (20.6%) were mild, 104 (26.1%) were moderate, and 170 (42.7%) were severe, whereas 18 (4.5%) were critical at admission. A total of 21.9 percent of the 188 patients with worsening symptoms had chronic pulmonary disease (COPD), 19.6 percent had diabetic mellitus, and 17.8 percent had asthma (Figure 1). More than half of the patients (59.3%) had comorbidities, with diabetic mellitus (28%) being the most frequent chronic condition, followed by COPD (17.1%) and hypertension (16.1%). Forty (10%) of the patients were treated in the ICU and 250 (66.8) received intranasal oxygen care. The average length of stay was 13 (SD: 5.7) days (Table 2).

### 3.3. Patient Treatment Outcome

Among 398 COVID-19 patients, 337 (84.7%) had favourable treatment outcomes, while (2.8%) transferred out and (12.5%) died in the treatment center (Figure 2).

### 3.4. Factors Associated with Poor Treatment Outcome of COVID-19 Patients

Variables like age, sex, residency, comorbidities, and admission status were statistically associated with poor treatment outcomes in bivariate logistic regression. When compared to their counterparts, the odds of poor treatment outcome among COVID-19 patients were significantly higher among COPD (AOR = 5.62; 95% CI: 2.49–12.70), asthmatic (AOR = 2.8; 95% CI: 1.17–6.67), CKD (AOR = 4.81; 95% CI: 1.27–18.22), diabetic mellitus (AOR = 2.27; 95% CI: 1.02–5.09), and HIV positive (AOR = 10.44; 95% CI: 3.0–36.35). Furthermore, people aged 55 and above years old (AOR = 4.35, 95% CI: 1.30–14.60) were nearly four times more likely to have poor treatment outcomes compared to 0-24 years. On the other hand, patients who were in severe or critical conditions during admission were 3.73 times more likely to have poor treatment outcomes (AOR = 3.73, 95% CI: 1.17–11.95) (Table 3).

## 4. Discussion

The COVID-19 pandemic is a worldwide public health issue that has resulted in increased anxiety, death, and deterioration of health in people with comorbidities and the elderly [24, 25]. In this study, we found that 15.3% of COVID-19 patients had poor treatment outcomes, which is similar to the report from Wuhan Pulmonary Hospital (11.73%) [26] and higher than Ethiopian findings (1.9%) [27]. On the contrary, this study's poor treatment outcome was lower than that of Belgium (29.9%) [28] and China (28.27%) [29]. These disparities could be the result of differences in care quality, sample size, age, comorbidities, study time, and settings. We discovered that the likelihood of a poor treatment outcome rises with age. Older patients were more likely than younger patients to have poor treatment results, according to studies from China [13, 29–32], Kurdistan [33], Saudi Arabia [34], and England [35]. This could be related to the body's immune defense system deteriorating with age, and older persons were more prone to severe disease and poor treatment outcomes from COVID-19 infection because they were more likely to have many chronic conditions that hampered their health [36].

Our study found that diabetic mellitus patients had higher odds of COVID-19 poor treatment compared to those without disease. Previous studies found that the presence of diabetes increased mortality in patients with COVID19, which was consistent with our finding [30, 33, 37–39]. Individuals with COPD, and asthma, had also considerably worse treatment outcomes than those who did not have the disease (*p* < 0.05). This is consistent with a study from Italy [40], and China [26, 30, 41], Germany [42], and Saudi Arabia [34], which found that patients with heart disease, asthma, and COPD had a poor COVID-19 prognosis. In addition, HIV positive and CKD COVID-19 patients had higher odds of poor treatment outcome compared to their counterpart. These could be due to patients with these comorbidities are more prone to acquire a more severe health condition and disease development, increasing their susceptibility to bad outcomes [43].

In this study, when compared to their counterparts, patients with severe/critical conditions during admission were more likely to have poor treatment outcomes. The study from China [44] and India [45] also reported the same trends among patients with worsening health conditions during admission. This can be explained by the fact that persons who were in those situations may have a chronic illness that worsens their health and leads to poor treatment outcomes. Even though we evaluated patients' treatment outcomes in a health center that served patients from 28 different districts, our study had significant limitations. First, because the data for the study was gathered from secondary sources, incomplete patient information posed a significant barrier. Second, due to the retrospective nature of the study design, all factors that were not available on registration were not included in the analysis. Moreover, the cross-sectional nature of the study design also does not indicate the cause and effect relationship between the factors.

## 5. Conclusion

In this study, we found that a significant number of patients had favourable treatment. Moreover, having complicated situations at admission, and chronic illnesses such as COPD, CKD, asthma, diabetic mellitus, and HIV/AIDS, participants were significantly associated with poor treatment outcomes. We found that respondents aged 55 and above years old were also associated with poor treatment outcomes. Therefore, critical follow–up and management of patients with underlying diseases and worsening health conditions during admission is required.

## Figures and Tables

**Figure 1:** General health status of the patients at admission compared by types of chronic illnesses.

**Figure 2:** Treatment outcome of Patients with COVID-19 at the treatment center in Arsi zone, 2021.

**Table 1:** Sociodemographic characteristics of COVID-19 patients admitted to the treatment center in Arsi zone, 2021.

Variable	Categories	Frequency (%)
Sex	Male	237 (59.5)
	Female	161 (40.5)

Age category	0-24 year	98 (24.6)
	25-34 year	91 (22.9)
	35-44 year	56 (14.1)
	45-54	52 (13.1)
	Above 55 years	101 (25.4)

Mean age	39 (SD: 19.4)	

Residence	Rural	247 (62.1)
	Urban	151 (37.9)

**Table 2:** Clinical characteristics of patients admitted with COVID-19 to the treatment center in Arsi zone, 2021.

Clinical characteristics	Categories	Frequency (%)
Clinical manifestation	Yes	374 (94)
	No	24 (6.0)

Co-morbidity	Yes	236 (59.3)
	No	162 (40.7)

Status	Asymptomatic	24 (6.0)
	Mild	82 (20.6)
	Moderate	104 (26.1)
	Severe	170 (42.7)
	Critical	18 (4.5)

Type of comorbidity	Hypertension	52 (16.1)
	Chronic cardiac disease	34 (10.6)
	COPD	55 (17.1)
	Asthma	47 (14.6)
	Chronic kidney disease (CKD)	14 (4.3)
	Diabetic mellitus	90 (28.0)
	Human immune virus (HIV)	15 (4.7)

Intranasal oxygen use	Yes	250 (66.8)
	No	124 (33.2)

Place of care	Ward	358 (90.0)
	ICU	40 (10.0)

Length of stay	Less than 15 days	263 (66.1)
	15 and above days	135 (33.9)
	Mean(SD)	13 (5.7)

**Table 3:** Bivariate and multivariate logistic regression analysis of factors associated with the treatment outcome of COVID-19 patients, 2021.

Categories	Treatment outcome		COR (95% CI)	AOR (95% CI)
	Favourable (%)	Poor (%)		
Age				
0-24 year	91 (92.9)	7 (7.1)	1	1
25-34year	85 (93.4)	6 (6.6)	2.12 (0.61,7.36)	0.83 (0.18,3.94)
35-44 years	49 (87.5)	7 (12.5)	3.95 (1.15,13.64)	1.06 (0.24,4.61)
45-54 years	43 (84.3)	9 (15.7)	4.16 (1.20,14.36)	2.64 (0.62,11.16)
55 and above years	69 (68.3)	32 (31.7)	4.77 (1.62,14.07)	4.35 (1.30,14.60)^∗^
Sex				
Female	137 (85.1)	24 (14.9)	0.95 (0.54,1.66)	1.14 (0.56,2.34)
Male	200 (84.4)	37 (15.6)	1	1
Residence				
Rural	132 (87.4)	19 (12.6)	1	1
Urban	205 (83. 0)	42 (17.0)	1.42 (0.79,2.55)	1.26 (0.62,2.57)
Hypertension				
Yes	40 (76.9)	12 (23.1)	1.82 (0.89, 3.71)	1.58 (0.68,3.69)
No	297 (85.8)	49 (14.2)	1	1
Chronic cardiac disease				
Yes	26 (76.47)	8 (23.53)	1.81 (0.78,4.20)	2.46 (0.85,7.09)
No	311 (85.4)	53 (14.6)	1	1
COPD				
Yes	32 (58.2)	23 (41.8)	5.78 (3.06,10.87)	5.62 (2.49,12.70)^∗^
No	305 (88.9)	38 (11.1)	1	1
Asthma				
Yes	32 (68.1)	15 (31.9)	3.11 (1.56,6.18)	2.80 (1.17,6.67)^∗^
No	305 (86.9)	46 (13.1)	1	1
CKD				
Yes	7 (50.0)	7 (50.0)	6.11 (2.06,18.11)	4.81 (1.27,18.22)^∗^
No	330 (85.9)	54 (14.1)	1	1
Diabetic mellitus				
Yes	73 (81.1)	17 (18.9)	1.27 (0.68,2.36)	2.27 (1.02,5.09)^∗^
No	264 (85.7)	44 (14.3)	1	1
Malignance				
Yes	10 (66.67)	5 (33.33)	2.92 (0.96,8.86)	2.29 (0.45,11.78)
No	327 (68.9)	56 (31.1)	1	1
HIV/AIDS				
Positive	6 (40.0)	9 (60)	9.55 (3.26,27.94)	10.44 (3.0,36.35)^∗^
Negative	331 (86.4)	52 (13.6)	1	1
Admission status				
No symptom/mild	102 (96.2)	4 (3.8)	1	1
Moderate	94 (90.4)	10 (9.6)	2.17 (0.72, 6.58)	2.14 (0.58,7.93)
Severe/critical	141 (75)	47 (25)	6.66 (2.56, 17.34)	3.73 (1.17,11.95)^∗^

Note: ^∗^*p* value < 0.05.

## Data Availability

The datasets supporting the conclusions of this article are included in the supporting information.

## Abbreviations

AIDS: Acquired immune deficiency syndrome
AOR: Adjusted odds ratio
CI: Confidence interval
CKD: Chronic kidney disease
COPD: Chronic pulmonary disease
CoVs: Coronaviruses
COR: Crude odds ratio
HIV: Human immune virus
HCoV: Human coronavirus
LMIC: Low and medium-income countries
ICU: Intensive care unit
MERS: Middle East respiratory syndrome
PCR: Polymerase chain reaction
OR: Odds ratio
SARS: Severe acute respiratory syndrome
SD: Standard deviation
WHO: World Health Organization.
